# The tumor patient in the COVID-19 pandemic–an interview-based study of 30 patients undergoing systemic antiproliferative therapy

**DOI:** 10.1371/journal.pone.0256047

**Published:** 2021-08-11

**Authors:** Ulrich Kaiser, Ursula Vehling-Kaiser, Jörg Schmidt, Ana Hoffmann, Florian Kaiser

**Affiliations:** 1 Clinic and Polyclinic for Internal Medicine III, Regensburg University Hospital, Regensburg, Bavaria, Germany; 2 Oncological/Palliative Network Landshut, Landshut, Bavaria, Germany; 3 Institute for Market Research in the Health Care System Munich, Munich, Bavaria, Germany; 4 VK&K Studien GbR Landshut, Landshut, Bavaria, Germany; 5 Clinic for Haematology and medical Oncology, University Medical Centre Göttingen, Göttingen, Lower Saxon, Germany; China University of Mining and Technology, CHINA

## Abstract

**Introduction:**

Five months after COVID-19 first occurred and protective regulations were introduced, patients at three outpatient hematological/oncological centers in Bavaria who had received antiproliferative tumor therapy (n = 30) were questioned about the pandemic’s impact.

**Patients, materials and methods:**

In recorded semi-structured telephone interviews, the patients answered questions about their quality of life, treatment procedures, their relationship with medical care staff and modern communication technologies. Each interview consisted of 28 questions. The average length of an interview was 30 minutes. The interviews were transcribed and analyzed by means of a qualitative content analysis according to Mayring.

**Results:**

The COVID-19 pandemic adds to the burden of patients by decreasing their social contacts. They perceived the new isolation and protective measures in outpatient clinics as mostly positive and said its impact had been only slightly adverse. With the implemented safety measures, they feel adequately protected and looked after and want their antiproliferative therapy to be performed as scheduled. Talking to medical staff provides additional reassurance.

**Conclusion:**

Although the COVID-19 pandemic has exacerbated the social isolation of tumor patients, it has had only a minor effect on tumor therapy in the surveyed patient population. The benefits of modern communication options to tumor patients remains uncertain and should be investigated further in future studies.

## Introduction

At the end of 2019, severe respiratory infections caused by the novel RNA beta coronavirus SARS-CoV-2 were identified in China for the first time. In January 2020, a first case of a COVID-19 infection was described in Germany, and in March 2020, after COVID-19 had spread worldwide, it was declared a pandemic [1]. COVID-19 can occur both in the upper and the lower respiratory tracts and elsewhere. When it occurs in the lower respiratory tract, in particular, it can lead to a severely impaired gas exchange, potentially with a fatal outcome. The risk group for a severe course of a COVID-19 infection includes people with comorbidities and a weakened immune system [2]. Tumor patients in particular belong to this risk group due to their malignant disease and the immunosuppressive side effects of antiproliferative therapies [3]. Compared to the remaining population, lung involvement increases in this patient group as does mortality [4, 5]. In addition, hypersensitivity pneumonitis, which occasionally occurs during antiproliferative therapy with checkpoint inhibitors, has a similar progression and a similar clinical picture as pneumonia caused by COVID-19 [6]. The COVID-19 pandemic has thus led to great uncertainty among patients regarding the benefit/risk ratio of antiproliferative therapies [7]. The German Society of Hematology and Oncology (DGHO) and the European Society for Medical Oncology (ESMO) have issued recommendations for safety precautions in the treatment of tumor patients with regard to COVID-19 infections, including the wearing of masks, checking patients before they’re allowed to enter treatment premises, banning relatives from entering, shortened times for interactions and the physical separation of patients (social distancing rules). In addition, they recommended the increased use of telemedicine and digital medicine [2, 8].

In summary, the COVID-19 pandemic represents a new and unprecedented situation for tumor patients undergoing antiproliferative therapy. As little was hitherto known concerning the personal and therapeutic consequences of the pandemic from the perspective of tumor patients, the present study was undertaken to investigate the issue by means of qualitative semi-structured interviews. Special consideration was given to potential effects on the tumor therapy, the perception of tumor patients regarding the required hygiene and protective measures, their relationship with medical care staff, and their experiences and ideas regarding telemedicine communication options.

## Materials and methods

Three hematological/oncological outpatient clinics in Bavaria established identical hygiene and protective measures at the onset of the COVID-19 pandemic to prevent COVID-19 outbreaks in the clinics. These included the introduction of a two-shift system, entrance checks according to a set protocol (including the recording of body temperature and symptoms typical of COVID-19), an entry ban for accompanying persons, social distancing rules throughout the entire outpatient clinic, personal hygiene measures, an obligation to wear masks (FFP2), regular surface disinfection and ventilation of the premises, shorter consultations as well as the increased use of contact by telephone and digital consultations.

In May 2020, all patients who had received intravenous antiproliferative therapy (chemotherapy, antibody therapy, angiogenesis inhibitors, immuno-oncology) at the three participating hematological/oncological outpatient clinics between 1 April 2020 and 7 April 2020 were invited to participate in a recorded telephone interview. For this purpose, a semi-structured interview guide consisting of 28 open questions was developed (Table 1). All participants were comprehensively informed about the study and written consent was obtained prior to each interview. The documentation and analysis were anonymous. The average interview length was 30 minutes. There was no time limit: the interviewees were given sufficient time to answer. The Institute for Market Research in the Health Care System Munich conducted the interviews in June and July 2020.

**Table 1:** Interview guide for tumor patients.

**Personal handling of the COVID-19 pandemic**	
Question 1	What is the first thing you think of when hearing the words ‘COVID-19 pandemic’?
Question 2	How do you personally manage during the COVID-19 pandemic?
Question 3	Who or what helps you most to cope with the COVID-19 pandemic?
Question 4	What do you worry about most regarding the COVID-19 pandemic?
**Impact of the COVID-19 pandemic on the disease**	
Question 5	How did the COVID-19 pandemic affect your tumor disease?
Question 6	Has the COVID-19 pandemic changed your personal attitude to the treatment of your tumor disease (e.g. affected the duration of therapy; triggered a discontinuation of therapy or the delay of treatments)?
Question 7	Do you feel left alone with your tumor disease during the COVID-19 pandemic?
Question 8	If yes: How does this become apparent?
	Support during the COVID-19 pandemic
Question 9	If no: Who helps you to cope with this?
Question 10	Do you think that the COVID-19 pandemic has negatively affected the treatment of your disease? If yes: How did this become apparent?
Question 11	Do you suffer from the lack of social contacts caused by the COVID-19 pandemic?
Question 12	If yes: What bothers you the most about the lack of social contacts? (Multiple answers possible)
Question 13	If yes: Contact with whom do you miss the most?
**Impact of the COVID-19 pandemic on contacts inside the practice**	
Question 14	Are you currently afraid to go to an oncological practice or a radiotherapeutic (radiologist’s) practice? If yes: What are you afraid of?
Question 15	Do you feel safe in the oncological practice where you are treated?
Question 16	If yes: What about the practice gives you a feeling of safety?
Question 17	If no: What would give you a feeling of safety in the oncological practice?
Question 18	To what extent have the procedures in the oncological practice changed for you as a result of the COVID-19 pandemic?
Question 19	If they have changed: Are these changes a burden for you?
Question 20	What is especially important to you when you come to a medical practice during the COVID-19 pandemic?
Question 21	Has your relationship to the attending oncologist changed? If yes: How?
Question 22	Has your relationship to the practice staff changed? If yes: How?
**Modern communication possibilities**	
Question 23	Have you been able to gain experiences with telecommunication options (telephone consultation, video consultation)?
Question 24	If yes: How was it for you, what kind of experience was it for you?
Question 25	If no: What is your attitude towards these modern forms of telecommunication?
Question 26	Do you think the communication options offered during the COVID-19 pandemic (telephone consultations, video consultations) are adequate?
Question 27	If no: What do you miss?
Question 28	In your opinion, is the use of these forms of communication (via phone or video consultation) likely to increase or decrease in the future?

The interview method was recorded, semi-structured, qualitative interviews via telephone. As this method is based on open conversations, it ensures an atmosphere where the interviewees can express any relevant opinions and thoughts relating to the topic, providing meaningful results typical of the respective target group [9–12]. In addition, the interviewer can ask directly if something is unclear, or elicit further important information about the topic by using supplementary questions.

The interviews were transcribed for further processing. The answers were analyzed using the qualitative content analysis method according to Mayring [9, 13]. This is a multi-stage, structured, reproducible analytical process whose steps include categorization, coding, re-evaluation and analysis of the interviews, thereby abstracting qualitative data systematically and transparently. After an initial review of the material, the interview questions were taken as the main categories. Subsequently, subcategories were formed for each main category by summarizing and identifying key topics. All the interview data were then sorted using the system of categories, and documented in tabular form (coding). In the process, the categories were constantly re-evaluated and adapted when new insights were obtained. Finally, the results were summarized and analyzed. In addition, literal statements (quotes) by the interviewees were used in the analysis in anonymized form, which highlighted the participants’ way of thinking and expressing themselves. To ensure interpersonal validity, four researchers conducted and discussed the analytical process.

The objective of the qualitative survey was to examine the following questions in more detail:

- Did the COVID-19 pandemic change the patients’ attitude to their tumor disease/tumor therapy?
- Did the tumor patients suffer from the lack of social contact caused by the pandemic?
- Has the relationship between the tumor patients and the care staff changed?
- Do the tumor patients feel safe in the hematological/oncological outpatient clinic?
- Do the changed procedures in the hematological/oncological outpatient clinic pose an additional burden for the tumor patients?
- What do tumor patients think of the modern communication options offered during the pandemic?

A proposal for the present study was submitted to the Ethics Committee in Munich, but no ethics vote was required.

## Results

Out of the invited tumor patients (n = 39), n = 30 (22 female, 8 male) participated in the interviews. The age distribution of the interviewees was as follows: 30–40 years, n = 4; 40–50 years, n = 4; 50–60 years, n = 11; >60 years, n = 11. Twenty-eight patients had solid tumors (breast cancer, n = 14; colon cancer, n = 2; rectal cancer, n = 1; gastric cancer, n = 2; bronchial carcinoma, n = 3; prostate cancer, n = 2; cholangiocellular carcinoma, n = 1; urothelial carcinoma, n = 1; ovarian cancer, n = 1; cervical cancer, n = 1), two patients had a malignant hematological disease (highly malignant lymphoma, n = 2).

### Patients’ concerns and changes in behavior during the COVID-19 pandemic

The 30 interviewed tumor patients spontaneously associated the term ‘COVID-19 pandemic’ with the fear of the disease/infection and the restrictions associated with the pandemic, such as ‘having to stay at home’, isolation and quarantine.

*Quote: ‘The COVID-19 pandemic has triggered fears in me. At the moment, it is very present and dominant in my daily life.’*

The term was also commonly associated with the realization that COVID-19 is a very serious and life-threatening disease. Nevertheless, 29 out of the 30 interviewees said that they were coping well with the pandemic: they adhered to the official rules, only left the house if necessary and observed the hygiene regulations such as wearing face masks, social distancing and disinfection.

Quote: *’Actually quite well*, *I stick to the rules*, *distancing and mask and actually have no problem with it*.*’*

*First and foremost*, patients feel supported by their families/relatives when coping with the COVID-19 pandemic.

Quote: *’My daughter and my strong personality*. *There are worse things*, *we are still doing well*. *We have something to eat*, *we have a roof over our heads*, *so what more do you want*. *What bothers me is that people are never happy*.*’*

Next on the list were the protective and hygiene measures and their personal attitude to the issue.

Quote: *’One mustn’t panic*, *mustn’t give up*, *one has to think positive*, *be careful*.*’*

Two patients spontaneously mentioned medical care as something that also helped them. Only two out of the 30 interviewees said that they did not need help coping with the pandemic. The greatest concern of tumor patients during the COVID-19 pandemic was the risk of infection, followed by the uncertainty of how long the pandemic would last, and the carelessness of people who did not comply with the rules. Only one of the 30 patients stated that they were not worried.

### Lack of social contacts is a problem

Two thirds of the interviewed tumor patients suffered from the lack of social contacts caused by the pandemic.

Quote: *’Yes*, *a little bit*, *of course*. *I am normally a very open person and this is something I do miss*. *I like to talk*, *I enjoy having social contacts*.*’*

In addition to the overall lack of contacts, the patients viewed the lack of interaction with family, friends and particularly grandchildren as the greatest restriction they faced. They also missed the lack of contact with family and grandchildren the most.

*Quote*: ’*Yes*, *it was hard in my private sphere*, *I have grandchildren*, *two relatively small ones*. *One of them I haven’t seen for 3 months now*. *This is hard because it is at that age that you build a relationship*.*’*

### Impact of COVID-19 on tumor therapy

Approximately one third of the 30 interviewees described the impact of the COVID-19 pandemic on their tumor disease as major, mainly due to the fact that the pandemic made social contacts even more difficult.

*Quote: ’You are even more restricted because the immune system is very weakened and so you have to be even more careful and simply avoid certain things.’*

*Quote: ’One couldn’t get so much help and encouragement from friends, or one really had to go through a very tough isolation, not leave the house for weeks, months, or only go for short walks.’*

Two thirds did not think that the pandemic had an impact on their disease.

*Quote: ’Ultimately, the pandemic had no impact, my operation was beforehand and my rehabilitation went ahead. Chemotherapy and radiation treatments also took place. Actually, there were no restrictions.’*

Twenty-nine interviewees stated that their attitude to their tumor therapy had not changed; they did not consider postponing or discontinuing their treatment and they felt well cared for by their specialist practice.

*Quote: ’No, my attitude hasn’t changed. I have always felt very well taken care of and looked after.’*

All 30 tumor patients reported that they did not feel left alone with their disease during the COVID-19 pandemic. They named family members and the attending specialists as almost equally important in providing support in coping with the pandemic.

*Quote: ’I have my family, but I also have an oncologist when I have questions. I was always able to go to the doctor, there was no restriction.’*

Twenty-eight respondents confirmed that the COVID-19 pandemic did not have a negative impact on their therapy. They received their regular treatments and medical appointments: everything went as planned. Two patients reported that the pandemic reduced the frequency or length of their medical consultations.

### Safety in the oncological practice

None of the 30 tumor patients were, or had been, afraid to go to an oncological practice. Oncological specialist practices closely observe the safety and hygiene regulations.

*Quote: ’The precautions start as soon as you arrive: the door is locked. You arrive, they ask you all the questions on the list, measure your temperature, disinfect the hands. Only a certain number of people at a time are allowed in the practice. They make sure that social distancing is observed, that’s really great.’*

*Quote: ’Yes, it’s all happening quite fast. They go for 1000% safety.’*

All 30 interviewees felt safe in the oncological practice where they were treated.

*Quote: ’It became clear that the doctor was really behind it, so that COVID-19 could not get into the practice, because as a cancer patient you are already seriously ill and if that was added, that would have fatal consequences. The strict social distancing rules provide safety, the requirement to wear a mask and everything like that.’*

The consistent adherence to the hygiene regulations and the social distancing rules in the oncological practices gave the interviewees their most important reason for an adequate feeling of safety.

*Quote: ’They make sure there is social distancing, there are no more than 3 people in the waiting room at a time, they all wear masks and make sure that everything is as it should be.’*

The check upon entering the practice, the very attentive and consistent practice staff and the care taken by always-accessible doctors also gave the interviewees a feeling of safety.

*Quote: ’With regard to COVID-19 and with regard to the disease, when you simply have a weakened immune system–that it is organized in such a way that there are only a few patients in the practice, that strict checks are in place before you enter so that nobody who has a cold can get in.’*

The patients mentioned the entry check as a first change in practice procedures due to the COVID-19 pandemic, followed by the requirement to wear masks and the social distancing rules.

*Quote: ’From the start, I could phone at any time of the day or night. The practice has precautionary measures in place: you only get in if you have no fever and answer their questions.’*

A third of the interviewees also mentioned the entry ban for relatives.

*Quote: ’I feel safe because the rules there are extremely strict. No relative is allowed in, only people with an appointment can come and then they are asked beforehand, there are 8–9 questions, how do you feel, where have you been, etc.’*

Four interviewees regarded the shorter waiting times in the practice as a positive change caused by the pandemic. For 26 patients, the changes necessary for the continuation of the practice during the pandemic did not pose an additional burden. For three patients, the obligation to wear a mask was a burden, and one patient mentioned that having to get up earlier for the treatment was a burden. Almost all patients (n = 29) consider the social distancing and the hygiene rules to be the most important safety measures when entering a medical practice.

*Quote: ’First of all, that there is really enough space, that not too many people are inside. That hygiene is ensured. People’s seats were disinfected in the oncological practice that is important after all.’*

The third point on the list of required safety precautions is the obligation to wear masks. Four interviewees considered the check upon entering the practice as a particularly important safety measure.

*Quote: ’The check upon entering, there’s an automatic door, then an employee looks at who’s standing there. Then the employee opens the door, then the employee has a questionnaire, it is always filled in, if you were there yesterday, you’ll fill it in again today.’*

### Care by doctors and medical staff

For 29 patients, the pandemic did not change their relationship with the attending hematologist/oncologist. One patient mentioned an even stronger trust as a positive change. For 27 tumor patients, their relationship to the practice staff did not change either. One patient mentioned the fact that the staff were even more attentive towards patients as a positive change. The close relationship to the medical staff contributed significantly to the patients’ feelings of safety.

Quote: *’The human touch that they have in the practice*. *The good contact to the nurse*, *to the doctor’s assistant*, *to the doctor*. *That just means safety*.*’*

Two patients pointed out disadvantages in patient care connected to the pandemic (change of staff, shorter consultations).

### Modern communication possibilities

Twelve tumor patients had used modern communication options such as telephone or video consultations, while 18 patients had not had this experience.

Ten of the patients with experience of telephone or video consultations described their experience as definitely positive.

*Quote: ’Yes, I always speak to my psycho-oncologist on the phone.’*

*Quote: ’When I got home from the hospital, they said so that I don’t get infected, there will be a phone conversation about how it went and how it will go on. I asked everything and they explained everything and all was well.’*

Two patients were critical because they felt overwhelmed by the situation *(quote*: *’Everything happened so fast’*) or because they missed the personal contact with their doctor. Out of the 18 patients who had not had any experience with modern communication options such as telephone or video consultations, nine were positive/open to this possibility, while seven interviewees were rather skeptical and said they preferred a personal interaction with the doctor.

*Quote: ’No, I want to talk to the doctor in person.’*

*Quote: ’It’s great, you don’t have to sit in the waiting room and wait, this works faster, the speed is crucial.’*

Two interviewees could not or did not want to give an opinion on this.

Nine out of the 30 patients found the communication options such as telephone or video consultations that were offered during the COVID-19 pandemic to be sufficient. Four others thought they were a good alternative to personal contact with the doctor.

Quote: *’Very positive really*, *everybody concerned saves time*, *so the doctor has more time for his patients in the practice and he also has more time during the video consultation*. *You can’t do everything by video*, *but you can do the normal consultations by video*.*’*

Twelve interviewees did not consider these communication options as sufficient, as they missed the personal contact, which offers more closeness and advantages from a patient’s point of view.

*Quote: ’Not particularly good, because I see a doctor on the screen and he sees me, but he doesn’t see me in real life, I’d say, and I could imagine that his diagnosis would suffer.’*

Five patients did not wish to comment, as they had not yet experienced a telephone or video consultation.

Twenty tumor patients assumed that the use of modern communication options such as telephone or video consultations would increase in future. Six patients thought that it would remain unchanged and four interviewees believed that the use of these communication channels would decrease.

## Discussion

The COVID-19 pandemic took patients and medical staff in Germany by surprise and resulted in significant changes to the procedures of oncological outpatient clinics due to the necessary hygiene and protective measures. Based on the interviews at hand, this study examined the consequences of the COVID-19 pandemic from the perspective of tumor patients.

The COVID-19 pandemic and the required general protective measures may lead to social isolation in tumor patients, who are particularly at risk of infection. However, personal attention is of fundamental importance to these patients in order to avoid serious consequential damage [14]. The interviewed patients felt especially affected by the decrease in contact with family members, despite already being familiar with medically required isolation measures as part of their usual antiproliferative therapy procedures. On the other hand, the patients felt adequately cared for by nursing staff despite the required social distancing rules in the outpatient clinics. In some cases, they even felt that they received more intensive care than before the pandemic. This personal contact seemed not only to promote trust, but also to counteract social isolation and have patients accept the safety regulations better [15].

In addition to suffering from the social isolation, many patients were afraid of getting infected. Nevertheless, all patients considered the risk of getting infected with COVID-19 at the oncology clinics to be very low. The new safety and hygiene measures contributed significantly to this and were considered necessary. The protective measures did not result in any greater burden to the patients.

While it was initially expected that more patients would discontinue treatment [16], the new safety precautions and hygiene regulations seem to have provided patients with a sufficient feeling of safety to avoid discontinuation of their antiproliferative therapy. This is in line with the results of a survey of gynecological patients in May 2020, who wanted to continue their tumor therapy despite an increased risk and the fear of an infection with COVID-19 [17]. DGHO also considers that the benefits of meaningful and planned chemotherapy are higher than the risks of COVID-19 infection [2].

Besides family members, the attending hematologists/oncologists played an important role in helping patients cope with the COVID-19 pandemic. This underlines the need for regular doctor-patient contact within the pandemic-related restrictions [17].

Modern communication methods (e.g. telephone contact with the patients) could provide a solution to this, as recommended by minimizing contacts, as recommended by hematological/oncological professional societies [2, 8]. About half of the interviewed patients considered digital communication to be very helpful in some ways, and to be practicable during the pandemic. Although most of the patients assumed that the use of modern communication channels would increase in the future, about one third of the patients did not consider them to be an adequate substitute for a personal conversation.

This is somewhat in contrast to N. Meti et al., who consider a return to pre-pandemic personal patient care unlikely [18]. However, tumor patients are a highly sensitive group of patients for whom personal conversation with their doctor is a cornerstone of therapy [19, 20].

The results of the interviews indicate that older patients in particular are more critical of the possibilities of telemedicine. This is in line with the results of Cindy Y. Jiang et al., who were able to demonstrate that while telemedicine can be used successfully in patients of the older generation, it still poses many challenges [21].

Considering the opinions expressed by the patients and the small number of studies [22], it becomes clear that further studies on the use and benefit of modern communication media–as S. P. Hasson et al. have already demanded for the inpatient sector [23]–are also urgently needed for the outpatient care of tumor patients [24].

## Limitations

The survey was conducted in a rural area, which is characterized by intensive doctor-patient contact and an under-representation of internet and telemedicine communication due to a common lack of communications infrastructure. The results of a similar survey may differ if it was conducted in a large city. Only patients who were being treated in oncological outpatient clinics at the time, participated in the interviews. Patients who stayed away from outpatient clinics were not included. This could limit the significance of the question about COVID-19-related therapy discontinuation [15, 25]. Nevertheless, the collected data show that at least some of the tumor patients were motivated and willing to continue antiproliferative therapy during the pandemic with appropriate safety measures. Moreover, the survey took place at a time when infection rates were low in Germany. Especially in times of increasing infection numbers, the statements, particularly concerning safety and hygiene measures, are significant.

## Conclusions

It has been possible to continue the treatment of tumor patients during the COVID-19 pandemic to the satisfaction of the patients by consistently adhering to safety precautions also in outpatient settings. Conversations with doctors and nursing staff are essential for the patients, especially during the crisis situation with its contact restrictions, and such interactions should be maintained as far as possible. The addition of telemedicine media could play an important role in this in the future.
